RETRACTED

# Strategies for Ideological and Political Education in Colleges and Universities Based on Deep Learning

**DOI:** 10.1155/2022/5322677

**Published:** 2022-09-26

**Authors:** Ying Sun

**Affiliations:** Jilin Animation Institute, Changchun, Jilin 130012, China

## Abstract

Ideological and political education in colleges and universities is routinely burdened with the job of building morality and cultivating people, which is related to the cultivation of college students' ideals and beliefs, spiritual pursuits, and political literacy. Based on self-determination theory (SDT), this paper modeled different learning motivations in the early stage of ideological and political courses and analyzed the learning motivation of different student groups combining the Gaussian mixture model (GMM) and stacked autoencoder (SAE). Meanwhile, the study in this paper compared the participation characteristics of different learning motivation clusters, the differences between the ideological and political course performances of students with different learning motivations, and the potential link between learning motivation and learners' educational level. The experimental results show that students with extrinsic motivation will have better performance in the courses. The strength of extrinsic motivation is positively correlated with students' academic performance, and 70% of students with intrinsic motivation achieve excellent results. In addition, the *χ*^2^ test result of the two courses selected is 6.442, which confirms the effectiveness of the clustering model proposed in this paper from the side and provides effective theoretical support for the implementation and reform of ideological and political education strategies.

## 1. Introduction

As information technology increasingly modernizes, tremendous changes have taken place in people's lives, and various fields such as politics, economy, and culture have all taken the express train of the information age to move forward. In recent years, with the gradual entry of information technology into the field of education, more and more education researchers have devoted themselves to the practical exploration of the deep integration of information technology and subject teaching [1]. The integration of information technology into the ideological and political teaching of colleges and universities will inevitably bring new opportunities and challenges to the education system [2].

At present, online education has become a hot issue and the optimization of online education service quality has gradually become common demand of social life. E-learning has gained enormous popularity due to the accessibility of various e-learning platforms such as Moodle, Blackboard, MOOC, and so on [3]. Learning management systems such as MOOC and Moodle are widely used in enterprises, universities, and educational institutions, which offer certain advantages to the teaching of modern education. Online education is a computer-based learning environment in which students can freely choose learning materials and control their own learning pace, and students' ongoing learning behavior will be recorded in log files without interrupting their learning process. Through in-depth analysis of log files, students' learning behaviors can be studied qualitatively, which can provide useful information for teachers to improve instructional design. Many studies have shown that online learning has a significant impact on students' autonomous learning and knowledge acquisition [4]. For example, Liu and Yuan found that students can only learn effectively when they are highly motivated in networking activities. Different learning motivations produce different learning outcomes [5]. Firat et al. used the IMeL questionnaire method to determine the level of intrinsic motivation of open and distance education students [6, 7], and Dunn used the questionnaire method to classify learning motivation, which is used as an engagement indicator to predict students' final performance at the same time [8, 9]. However, not every student can benefit from an online learning model even if they enroll in the same courses, as learning outcomes are greatly influenced by students' self-regulated learning ability and motivation. In other words, learning motivation drives learning behavior, and learning behavior is an external manifestation of learning motivation and an important basis for evaluating the state of learning motivation. Differences in students' learning motivations will directly differentiate learning strategies selected. So, a high interest may be required for students' initial learning. With interest, students' curiosity will be stimulated, and students' motivation to learn will be enhanced. Different learning participants have different learning motivations and goals; the motivation may not be just to get better grades or certificates, it may be that they are interested in a particular chapter or forum, which will support them to communicate with more like-minded scholars. Therefore, it is urgent to better understand the inner relationship between students' learning behavior, final performance, and learning motivation. To gain a more objective understanding of the relationship between learning motivation, engagement, and final performance, different learning motivations can be measured by analyzing online learning behavior data. Currently, online learning is often lacking in guiding students' learning depth. Improving the depth of learning depends on the user experience on the online learning end of the learners and the reinforcement of learning motivation. However, it is not easy to evaluate students' learning motivation and identify their differences in detail. In the traditional offline classroom environment, teachers can relatively easily grasp the specific situation of students' learning motivation through face-to-face interaction, while in the online learning environment, teachers must obtain this information through the information recorded by the learning platform. In addition, students with different educational backgrounds are able to enroll in the same course according to their own will, which leads to a huge number of participants in a given course, so it is indispensable to develop a method that can automatically detect various motivation types from large datasets.

RETRACTED

Although there have been some previous studies on learning motivation [10, 11], most of them are based on questionnaires, self-reports and interviews, and other data for analysis, and few use data collected from online learning platforms, which makes the analysis process very labor-intensive, and the final analysis results are too subjective. Even though there are some studies on online learning behavior, these studies are based on the analysis of students' overall performance in the whole course semester, and the final research results cannot be fed back to the current course in time. According to the above problems, this paper attempts to process a large amount of information (demographic information and clickstream data) generated in the ideological and political education of colleges and universities through the method of machine learning (deep learning) and combines corresponding models and theories (self-determination theory, Gaussian mixture model, and deep coding automatic model) to clarify the relationship between learning motivation and external performance of students' ideological and political education. At the same time, it also provides relevant constructive suggestions for the implementation and reform of ideological and political education strategies.

## 2. Models and Methods

### 2.1. Self-Determination Theory

Self-determination theory (SDT), one of the most comprehensive and empirically supported theories about motivation [12], describes the learning motivation in the online learning environment in detail. Deci and Ryan defined SDT as an experience-derived theory of human motivation and personality in social settings that distinguishes motivation from autonomy and control. Related studies have shown that SDT has made an important contribution to the determination of students' motivation in an online environment [13].

RETRACTED

### 2.2. The Basic Principle of Gaussian Mixture Model Algorithm

#### 2.2.1. Related Concepts of Gaussian Mixture Model

The Gaussian mixture model (GMM) is a model composed of multiple Gaussian distributions, and the basic Gaussian mixture model adopts the method of linear superposition [14]. It assumes that the dataset consists of multiple potential clusters that conform to a Gaussian distribution, and that the final stacking result is the distribution presented. Although in general, the same dataset may contain different types of distributions, considering that the model is represented by a mixture of multidimensional Gaussian probability models, it can still fit any type of probability distribution.

Supposing that a random variable *X* is a mixture of *M* Gaussian distribution models, the Gaussian mixture model can be represented as follows:

(1) $$\begin{array}{c} P\left(x|\theta \right)=\overset{M}{\underset{m=1}{\sum }}\alpha_{m}\phi \left(x|\theta_{m}\right)\text{,} \end{array}$$

where *α*_*m*_ represents the weight of the *m*th Gaussian distribution in the Gaussian mixture model. This parameter is generally not given and satisfies the following formula:

(2) $$\begin{array}{c} \overset{M}{\underset{m=1}{\sum }}\alpha_{m}=1,\left(\alpha_{m}\geq 0\right)\text{.} \end{array}$$

Although it is generally impossible to know the components occupied by each Gaussian distribution in the mixture model, considering that the Gaussian mixture model is formed by the linear superposition of *m* Gaussian distributions, the sum of the weights of its constituent members is defined as 1. In formula (1), *ϕ*(*x|θ*_*m*_) is the probability density function of the *m*th submodel in the mixture model, Gaussian density function is the most used function, and *θ*_*m*_ can be represented by *θ*_*m*_=(*μ*_*m*_, ∑*m*), so *ϕ*(*x|θ*_*m*_)can be expressed by

(3) $$\begin{array}{c} \phi \left(x|\theta_{m}\right)=\frac{1}{\sqrt{2\pi \sum_{m}}}\exp\;\left\{-\frac{{\left(x-\mu_{m}\right)}^{2}}{2\sum_{m}}\right\}\text{,} \end{array}$$

where *μ*_*m*_ represents the mean of the *m*th Gaussian distribution component and ∑*m* represents the covariance matrix of the *m*th Gaussian distribution component.

Given that a Gaussian model can be determined by the probability density function and the parameter set *θ*, the parameter calculation of the hybrid model proposed in this paper uses the log-likelihood function of the maximization model to find the optimal sample parameters that make the cluster close to the actual distribution of the sample as far as possible, so as to obtain better performance clustering results. Equation (4) is a likelihood estimation function that calculates the key parameters of the sample dataset.

(4) $$\begin{array}{c} L\left(\theta \right)=L\left(X_{1},X_{2},\cdots X_{m};\theta \right)=\overset{m}{\underset{i=1}{\prod }}P\left(X_{i},\theta \right) \end{array}$$

where *X*_1_, *X*_2_, ⋯*X*_*m*_ represents the data samples of the model, *P*(*x*, *θ*) represents the probability density function of the model, and *θ* represents a vector consisting of one target parameter or multiple parameters to be estimated.

RETRACTED

Considering the hidden variables in the sample set, the process of directly using the maximum likelihood estimation method to estimate the model parameters will be quite tedious, and the optimization process will be quite long [15]. Therefore, the implicit variables need to be represented first. After determining the hidden variables, the maximum value of the likelihood function is obtained and after taking the logarithm of formula (4), formula (5) is the result obtained.

(5) $$\begin{array}{c} L^{\left(1\right)}\left(\theta \right)=\overset{m}{\underset{i=1}{\sum }}\;\log\;p\left(x_{i},\theta \right)=\overset{m}{\underset{i=1}{\sum }}\;\log\underset{Z_{i}}{\sum }p\left(x_{i},z_{i},\theta \right)\text{.} \end{array}$$

#### 2.2.2. Expectation-Maximization Algorithm

The expectation-maximization (EM) algorithm was first proposed by Dempster et al. EM algorithms are widely used in many algorithms in machine learning [16, 17] such as the parameter estimation in the K mean, the support vector machine (SVM) [18], the GMM, the hidden Markov model (HMM) [19], and the subject generation model (latent Dirichlet allocation, LDA) [20]. The EM algorithm refers to the iterative solution of some target parameters using a strategy of great likelihood estimation in all datasets, including hidden variables. The iteration of the EM algorithm is mainly done by two steps: the expectation Step and the maximization Step. The expectation step of the expectation-maximization algorithm is to calculate the expectation of the model according to the hidden state of the model, compute the Gaussian distribution of the guessed hidden data, and then fix the model parameters and use the maximum likelihood estimation to calculate the complete data including the observed data and the hidden data in sequence, which will finally obtain the parameters of the Gaussian mixture model. By that analogy, M steps are performed. Then, through iterating E step and M step, that is, adjusting the model according to the parameters (E step) and then adjusting the parameters according to the model (M step), the E step and the M step are alternately performed until the parameters of the solved Gaussian mixture model do not change substantially. Meanwhile, the algorithm achieves convergence and obtains the optimal expectation of the Gaussian mixture model, the covariance matrix, and the weights of each Gaussian distribution. The expected value of the log-likelihood function of the mixed model can be described by the initial values of the model parameters that have been selected, and the specific definition is

(6) $$\begin{array}{c} E_{Q}\left[\log\;p\left(\theta |Y,Q\right)|\theta^{\left(i\right)},Y\right]=\int \log\;\left[p\left(\theta |Y,Q\right)\right]p\left(Q|\theta^{\left(i\right)},Y\right)dQ\text{,} \end{array}$$

where *Q* represents the implicit data that cannot be observed and *θ*^(*i*)^ represents the posterior standard deviation after the *i*+1th iteration. The conditional expectation probability of the joint distribution of the mixture model can be expressed by

(7) $$\begin{array}{c} L\left(\theta ,\theta_{i}\right)=\overset{m}{\sum }\sum P\left(z_{i}|x_{i},\theta_{j}\right)\log\;P\left(x_{i},z_{i}|\theta \right)\text{.} \end{array}$$

The constraint of the maximum value of the log-likelihood function parameter under the conditional probability can be expressed by

(8) $$\begin{array}{c} \theta^{j+1}={argmax}_{\theta }L\left(\theta ,\theta^{j}\right)\text{.} \end{array}$$

Continue to iterate the above E step and M step and end the iteration when *θ*^(*i*)^ and *θ*^(*i*+1)^ are infinitely close.

RETRACTED

### 2.3. Deep Autoencoding Model

#### 2.3.1. Autoencoder

Autoencoder network belongs to a kind of neural network structure under unsupervised learning classification, which usually consists of three layers [21]. The ideal goal of an autoencoder network is to reproduce the original input data. Similar to the Seq2Seq model in natural language processing, an autoencoder network usually consists of two parts: an encoder and a decoder. Among them, the goal of the encoding network is to convert the relatively high-dimensional original input data into an encoding vector in a low-dimensional space, while the role of the decoding network is the opposite, which is to restore the low-dimensional vector to the data representation of the high-dimensional space [22].

The encoder consists of an encoding function *f*_*θ*_, and for each input data *x*, the encoding function can be expressed by

(9) $$\begin{array}{c} h=f_{\theta }\left(x\right)=f_{\theta }\left(\omega x+b\right)\text{,} \end{array}$$

where *h* is an intermediate vector obtained after the input data *x* are encoded by the encoder in the hidden layer, which can also be called an encoding vector. In the same idea, the decoding network is composed of a decoding function *g*_*θ*′_ that is, the decoder, which remaps the intermediate vector *h* from the low-dimensional space to the high-dimensional space, as shown in the following formula:

(10) $$\begin{array}{c} \hat{x}=g_{\theta^{\prime }}\left(h\right)=g_{\theta^{\prime }}\left(\omega^{\prime }h+b^{\prime }\right)\text{.} \end{array}$$

As shown in formula (11), the parameters *θ* and *θ*′ in the encoding stage and the decoding stage are obtained by continuously adjusting and updating to minimize the reconstruction error. . The essential principle of the autoencoder is to minimize the reconstruction error$L\left(x,\hat{x}\right)$of the samples for M training sample data sets, which is often used to measure the difference between the input data *x* and the output data $\hat{x}$. To sum up, the specific definition is shown in the following formula:

(11) $$\begin{array}{c} \phi_{AB}\left(\theta ,\theta^{\prime }\right)=\frac{1}{M}\overset{M}{\underset{m=1}{\sum }}L\left(x,g_{\theta^{\prime }}\left(f_{\theta }\left(x^{m}\right)\right)\right)\text{.} \end{array}$$

Both the encoder and the decoder are implemented by nonlinear mapping, and their specific definition is shown in equations (12) and (13), where *s*_*f*_ represents the activation function of the encoding stage and *s*_*g*_ represents the activation function of the decoding stage. The parameter set of the encoder can be represented as *θ*={*W*, *b*}, and the parameter set of the decoder can be represented as *θ*′={*W*^*T*^, *b*}, where *b* and *d* both represent bias vectors and *W* and *W*^*T*^ represent weight matrices.

(12) $$\begin{array}{c} f_{\theta }\left(x\right)=s_{f}\left(Wx+b\right)\text{,} \end{array}$$

(13) $$\begin{array}{c} g_{\theta^{\prime }}\left(x\right)=s_{g}\left(W^{T}x+d\right)\text{,} \end{array}$$

(14) $$\begin{array}{c} L\left(x,\hat{x}\right)={\left\|x-\hat{x}\right\|}^{2}\text{.} \end{array}$$

RETRACTED

#### 2.3.2. Deep Feature Learning

The deep learning network model is to input the original input data into a neural network with multiple hidden layers. After the nonlinear operation of multiple hidden layers in the middle, the final output of the hidden layer is the same as the input data through the deep network model. The deeper it learns, the deeper the features are abstracted [23]. However, some datasets do not have initial labels, and deep feature learning is divided into three categories based on whether the initial labels are involved in the entire network training process, namely, supervised feature learning, semi-supervised feature learning, and unsupervised feature learning. Among them, supervised feature learning can be called classification. Semi-supervised feature learning is between supervised feature learning and unsupervised feature learning, referring to the existence of labeled data and unlabeled data in the training data. Unsupervised feature learning is also called clustering [24].

### 2.4. Experimental Data

#### 2.4.1. Data Selection

The datasets used in this study were collected and curated by researchers at the Open University and relevant content and materials for courses were delivered through a virtual learning environment (VLE). Hereby, we extracted two different courses A and B on ideological and political education from this platform for research.

#### 2.4.2. Data Preprocessing

The original clickstream data of students collected from the Open University Learning Analysis Dataset (OULAD) were used as features for analysis. Since there are some redundant features in the original feature set, we removed these features, filled in the missing values, and analyzed certain features in sequence. Then, the existing features were summed and averaged to characterize the available learning into four categories: demographics, interaction behavior, registration information, and evaluation information. In terms of data selection, we selected two representative courses in the Open University in 2018 and 2019. The selected course presents more than 300 students with at least two lesson videos in the course and a large number of students in the course who failed their final grades. For all courses that meet these criteria, we have selected courses A and B, with a total of 846 students in the selected courses. Finally, we anonymized the data in accordance with the ethical and privacy requirements applied in the Open University.

## 3. Experimental Results and Analysis

### 3.1. Analysis of Different Learning Motivation Clusters and Learning Behavior Characteristics

This article used two courses, A and B, to examine the association between motivation, student engagement, and final performance. After preprocessing the data, a total of 744 students enrolled in these two courses, with 363 enrolling in course A and 381 enrolling in course B. In order to determine the motivation level of students as early as possible based on the interaction data and demographic information of the virtual learning environment, we used the interaction data before the first job submission. In Table 1, we calculated the distribution of final grades for students in both courses who did not submit their first assignment.

According to Table 1, if a student does not submit their first assignment, the probability of failing the course is greater than 90% (withdrawing is also considered a failure), making first assignment submission an important factor in final grade prediction. However, considering that students' learning motivation is largely determined by their demographic information, simply submitting the first assignment is not sufficient to understand the different behavioral patterns of students for the purpose of predicting learning motivation, and their behavioral data and learning styles recorded in the online learning platform system shall prevail. To this end, we integrated and analyzed students' behavioral data, demographic information, assessment quiz information, and course registration information recorded by the virtual learning environment before submitting the first assignment, such as Homepage Clicks, Average Clicks, Forum Clicks, and so on. This article kept all the details of this information in the virtual learning environment.  Table 2 shows the characteristics and associated descriptions used in this study.

RETRACTED

This section examines the quantitative statistics of relevant features in each of the different learning motivation classes and compares these feature values in the same group. This article described the level of participation of each variable in different categories by mean (Mean) as well as standard deviation (Std).  Table 3 describes the differences in indicators of different characteristics of each group. As you can see from the table, Avg delay represents the level of procrastination of students in different motivation groups, and the results show that students in the IMFS and UMS groups are more likely to delay submitting assignments than the remaining two groups. The larger values for the standard deviation of the two groups of students (Std = 12.11 and Std = 10.37) indicate that the two groups of students are weak in time management and control of learning systems. Conversely, students in the IMPS and EMS groups have nearly the same standard deviations, which are (Std = 8.91 and Std = 8.23), indicating that students in the two groups always submit assignments at similar times or study at a fixed rate. In the first job, the average scores for IMPS group, IMFS group, EMS group, and UMS group are Mean = {70.55, 65.72, 79.91, 71.87}, respectively. It can be found that students in the UMS group have a higher average score than students in the IMFS group, indicating that students in the UMS group work harder than students in the IMFS group from the beginning of the course to the submission of the first assignment, with higher grade point averages and higher assignment scores. However, it is also concluded that students in the UMS group are more likely to delay submitting assignments, and as course content becomes more complex, their interest in learning is more likely to be affected. For students in the EMS group, they scored the highest average on their first assignment and studied at a relatively stable pace during this time. These quantitative and other data analysis results are consistent with our previous analytical modeling of learning motivation. Compared with using deep learning algorithms to analyze multidimensional clickstream data and cluster different learning motivations, it is more explanatory to analyze different learning motivation groups from statistical dimensions.

RETRACTED

### 3.2. Experimental Results and Analysis of Learning Motivation Clustering Model Based on GMM and SAE

In this section, we compared the relationship between the clustering results of learning motivation and students' final grades to verify our clustering results, and the final clustering results of different learning motivations are shown in Figure 1. The relevant clustering results are usually hierarchical or partitioned, and partitioning makes it easier to show each cluster in a 2D plot rather than a dendrogram, so this paper used the partition method to display the final clustering results. These components are calculated based on the maximum possible variance of the variables used in order to show as many defects as possible in the data.

It can be seen from Figure 1 that the clustering results of the cluster scatter diagram of learning motivation and students' final grades are roughly divided into three groups, and there may be a small amount of overlap between these clusters. Among them, the black clustering can be interpreted as a class of groups with extrinsic learning motivation. These students have strong learning goals and objectives, and most of them are rewarded or certified for high scores. In addition, the extrinsically motivated group is the largest group, and most participants in this group completed the course, with most of their final grades tending to be above 80 and very few students failing their course. This is consistent with the definition of extrinsic learning motivation as explained. In contrast, most of the students in the red clustering have less than 60 points in their academic performance, and the number is smaller than that of the black class. This may be due to the fact that some of this group of students do not have final grades, and the ultimate goal of them is not to get high grades or to get an award certificate, whereas they may be interested in a certain knowledge point or want to discuss and exchange with other scholars in the forum of the learning website. We call them intrinsically motivated students. The learning behavior of this group of students is often driven by intrinsic motivations such as emotion, interest, or temporary curiosity and is rarely affected by external motivations. Most of the students with cyan dots in the figure have no grades and no obvious distribution rules. We classify them as students with other motivations or no obvious motivations. This group of participants is less active on online learning platforms. Only a small number of students' final results are counted, and the attrition rate is very high, which is the smallest group among the three groups.

RETRACTED

### 3.3. Influence of Intra-Cluster Error Variance and Silhouette Coefficient on Model Performance

Since the learning features analyzed do not belong to the previously defined categories, this study used internal evaluation indicators to analyze the performance of the clustering model. In order to determine the optimal number of clusters for the clustering results, this section uses the error variance within the cluster and the silhouette coefficient to verify the reliability and validity of the clustering results, and the results are shown in Figure 2. The intra-cluster error variance (SSE) is used as the performance index [25]. The smaller the index value is, the higher the convergence degree of each cluster is. However, the value of intra-cluster error variance (SSE) is not as small as possible because there is an extreme case that all sample points are regarded as a cluster, in which the error variance within the cluster is 0, and the final classification effect is obviously not achieved. Therefore, it is necessary to seek a balance between the number of clusters and the variance of intra-cluster error variance (SSE). The elbow method solves this balance problem [26]. Assuming that there is an initial value K, we defined it as the largest possible number of clusters and then incremented the number of clusters from 1. In fact, the data have an underlying pattern, that is, there is a real optimal number of clusters, and when the number of clusters set by the model continues to approach this value, the intra-cluster error variance (SSE) will decrease rapidly. However, when the number of clusters set exceeds the actual optimal number of clusters, the rate of decrease of the intra-cluster error variance will become slow. By analyzing the changes in the value of the descending derivative, the final optimal cluster can be determined.

In general, the higher the average silhouette coefficient, the better the quality of the clusters. From the average silhouette coefficient in the above figure, the optimal number of clusters should be 2 clusters, and the value of the average silhouette coefficient is the highest at this time [27, 28]. However, according to the elbow rule, when *k* = 2, the correlation curve of the intra-cluster error variance (SEE) is not a rapidly decreasing trend. In other words, it is not an inflection point when *k* = 2. But when *k* = 3, the value of intra-cluster error variance (SEE) will drop sharply, which is an inflection point, and the value of the average profile coefficient is also relatively high at this time, only slightly lower than the value at *k* = 2. Therefore, when comprehensively analyzing the average silhouette coefficient and intra-cluster error variance, *k* = 3 is the best choice for the number of clusters. The final clustering results obtained in this paper are consistent with the type of motivation defined by SDT theory, which indirectly proves the rationality and interpretability of this method. The influence of intra-cluster error variance (SSE) and silhouette coefficient on the optimal number of clusters is shown in Figure 2.

RETRACTED

### 3.4. The Correlation Experiment between Learning Motivation and Educational Level

Except for the above, this paper also analyzes the relationship between different educational levels and learning motivation. In this dataset, the educational attainment of the participants is broadly classified into 4 categories: “A level or equivalent,” “higher education (HE) qualification,” “below A level,” and “postgraduate qualification.” Figure 3 shows the distribution of students with different educational levels in different motivation groups. As can be seen from the graph, students with “A grade or equivalent” and “below A grade” educational levels make up about 70% of the student body. In the group of students with extrinsic motivation, the distribution of students of the four education levels is relatively even. In the group of students without obvious motivation (no motivation), students with “higher education (HE) qualification” and “postgraduate qualification” educational levels account for a small proportion of the total students, which is in line with the fact that most of the students with higher educational levels will have strong learning motivation or learning goals.

Table 4 illustrates the chi-square test for different educational levels for different motivation groups, and the *χ*^2^ statistic tests the difference between the expected and true distribution of different educational levels for different motivation groups. Based on this, we used a table to calculate the *P* value, with *P* < 0.05 indicating that the null hypothesis is rejected, and there is a significant correlation between educational background and learning motivation. The parameter df refers to degrees of freedom, which represents the number of independent values that vary in the calculation. Because both course A and course B have 4 different educational levels and three different sets of motivations for learning, the degree of freedom is 6. According to Table 4, the *P* values for both courses are greater than 0.05. Therefore, it is concluded that there is no significant relationship between educational attainment and learning motivation, accepting the null hypothesis.

RETRACTED

## 4. Conclusion

By understanding the motivation for learning, it can help the reform of the ideological and political education system and methods of colleges and universities, and also help the teachers to better understand the learning progress and situation of the learners, so as to timely prescribe the right medicine according to the specific problems and intelligently intervene in different learners. On the basis of SDT, this paper analyzed and modeled different learning motivations in the early stage of the course. Meanwhile, the study in this paper compared the engagement characteristics of different learning motivation clusters, studied the differences of course performance between student groups with different learning motivations and the potential link between learning motivation and learners' educational attainment, and clarified the relationship between different student groups inside and outside the school and demographic information such as age distribution. The main conclusions are as follows:

1. The study proves that students' learning behavior is an important indicator to identify students' different learning motivations, and different learning motivations are significantly related to students' final ideological and political performance. Most of the students with intrinsic learning motivation have higher ideological and political academic performance, and some students with unclear motivation also have high academic performance. This may be related to other learning data not recorded outside the online learning platform, which can be further analyzed in future studies.
2. This paper proposes a deep clustering algorithm combining GMM and SAE based on the demographic information and clickstream data about learning behavior recorded in the Open University virtual learning environment. The optimal number of clusters is determined by two internal evaluation indexes of clustering experiments, that is, silhouette coefficient and intra-cluster error variance. The maximum value of the silhouette coefficient is 0.82, and the intra-cluster error variance is less than 1220 under the number of clusters from 2 to 14, with the minimum value of 198.
3. The deep clustering model proposed in this paper is compared with the clustering models in other papers, and a comparative study is carried out from multiple perspectives. The results show that the model greatly improves the accuracy of clustering results through in-depth analysis of clickstream data, and the statistical test values of *χ*^2^ in A and B courses are both 6.442, and the *P* values are only 0.371 and 0.349, respectively, which are greater than 0.05. The results further show that the model can more accurately analyze the learning motivation of different student groups and make up for the shortcomings in other clustering algorithms.

RETRACTED

## Figures and Tables

**Figure 1:** The relationship between clustering results and students' final scores.

**Figure 2:** The influence of intra-cluster error variance (SSE) and silhouette coefficient on the optimal number of clusters.

**Figure 3:** The distribution of educational level in different learning motivation groups.

**Table 1:** Final performance distribution for students who did not submit the first assignment.

Course	Withdrawn	Fail	Pass	Prob of failure
A	272	71	17	0.95
B	266	80	33	0.91

**Table 2:** Characteristics and description for learning analysis.

Learning characteristics	Signalment
Age	Learner gender
Highest education	Learner age
Region	The living areas of a learner when taking the course
Forum clicks	Number of times learner visits forums
Resource clicks	Number of times learner visits lecture notes and slides
Homepage clicks	Number of times learner visits the first page of a lesson
Average clicks	Average number of times learner visits different resources
Average delayed days	Average number of days delayed in submitting assignments
Final performance	Learner final performance
Activity type	This includes watching course videos, browsing websites, or quizzes
Date registration	The exact time students register for the course online
Assessment weight	Represents the weight of each assessment score in the student's final score
Assessment type	It could be a daily quiz, a midterm exam, or a final exam

**Table 3:** Characteristics and comparison of participation degree of different learning motivation groups.

Learning motivation	Avg clicks Mean/std	Resource clicks Mean/std	Score of the first assignment Mean/std	Avg delay Mean/std
IMPS	49.22/44.01	40.44/35.35	70.55/8.96	0.37/8.88
IMFS	25.56/19.78	19.87/13.61	65.72/13.09	3.43/12.11
EMS	87.81/65.98	80.21/59.42	79.91/7.89	2.44/8.13
UMS	86.12/59.98	80.36/60.87	71.87/10.94	8.23/10.37

**Table 4:** Chi-squared test for comparing different educational levels with different motivation groups in courses A and B.

Course	*χ* ^2^ test	df	*P* value
A	6.442	6	0.371
B	6.442	6	0.349

RETRACTED

## Data Availability

The dataset can be accessed upon request.
